The article "Upregulated periostin promotes angiogenesis in keloids through activation of the ERK 1/2 and focal adhesion kinase pathways, as well as the upregulated expression of VEGF and angiopoietin-1" was published in 2014. Journal: Mol Med Rep.

# Upregulated periostin promotes angiogenesis in keloids through activation of the ERK 1/2 and focal adhesion kinase pathways, as well as the upregulated expression of VEGF and angiopoietin-1

**DOI:** 10.3892/mmr.2014.2827

**Published:** 2014-10-31

**Authors:** ZHE ZHANG, FANGFEI NIE, XINLEI CHEN, ZELIAN QIN, CHUNFU KANG, BIN CHEN, JIANXUN MA, BOLIN PAN, YONGGUANG MA

**Affiliations:** Department of Plastic Surgery, Peking University Third Hospital, Beijing 100191, P.R. China

**Keywords:** periostin, fibroblast, keloid, endothelial cells, angiogenesis

## Abstract

Periostin, a secreted extracellular matrix protein, is highly expressed in wound healing and in various types of human cancer and is involved in angiogenesis. Keloids, considered dermal benign tumors, are granulomatous lesions characterized by capillary proliferation. However, the underlying regulatory mechanism of angiogenesis in keloids remains to be elucidated. The present study aimed to examine the effect of periostin on angiogenesis in keloids. The expression of periostin was upregulated and the vessel density was higher in human keloids compared with normal tissue, observed following staining with CD31 and CD105. Periostin demonstrated a markedly positive correlation with blood vessel density, which was assessed using CD31 staining (r=0.711; P<0.01) and a weak correlation was observed using CD105 staining (r=0.251; P<0.01). Conditioned medium from keloid fibroblasts (KFs) promoted the migration and tube formation of human umbilical vein endothelial cells (HUVECs) compared with normal fibroblasts and this effect may have been abrogated by the short hairpin RNA knockdown of periostin. Treatment with recombinant human periostin promoted the migration and tube formation of HUVECs by activating the extracellular signal-regulated kinase 1/2 and focal adhesion kinase signaling pathway. In addition, periostin increased the secretion of vascular endothelial growth factor and angiopoietin-1 in the KFs. In conclusion, these data suggested that upregulation in the level of periostin may promote angiogenesis directly and indirectly in keloids and may be a key factor in keloid development. Periostin may, therefore, be a promising therapeutic target in the treatment of keloids and other angioproliferative diseases.

## Introduction

Keloids and hypertrophic scars are two common proliferative lesions resulting from abnormal wound healing (1). Unlike hypertrophic scars, which are limited to the boundaries of the original wound and degenerate spontaneously, keloids, which are considered to be dermal benign fibroproliferative tumors, outgrow the original wound edges and invade the adjacent normal dermis, the regression of which over time is rare (2). Despite numerous available treatments, including excision, treatment for keloids remains ineffective due to their recurrence (3,4).

The article "Upregulated periostin promotes angiogenesis in keloids through activation of the ERK 1/2 and focal adhesion kinase pathways, as well as the upregulated expression of VEGF and angiopoietin-1" was published in 2014. Journal: Mol Med Rep.

At initiation, keloids are defined as granulomatous lesions characterized by capillary proliferation (5). The areas of angiogenesis in keloids may represent overproliferation of vascular granulation tissue in aberrant wound healing, in accordance with the pathology of keloids, which are characterized by an exuberant healing response (6). Several studies have suggested that angiogenesis and vascular factors are important in keloid progression, due to their prolonged erythematous period and invasive characteristics. In keloids, endogenous transforming growth factor-β1 (TGF-β1) and vascular endothelial growth factor (VEGF) promote angiogenesis (5,7,8). The levels of VEGF are upregulated and the levels of endostatin are downregulated in the sera and tissue of patients with keloids compared with normal controls, which may contribute to the imbalance in angiogenesis present in keloids (9). Upregulation in the notch signaling pathway also induces angiogenesis in keloids (10). Despite previous investigation of the angiogenic activity of keloids in previous studies, the underlying regulatory mechanism of angiogenesis in keloids remains to be elucidated.

Our previous study demonstrated that the expression of periostin is upregulated in keloids compared with hypertrophic scars and normal skin tissue (11). Periostin is a 90-kDa secreted extracellular matrix (ECM) protein, which is expressed mainly in collagen-rich, fibrous connective tissue (12). The upregulation of periostin has been observed in cutaneous wound healing, cutaneous fibrosis and in tumor progression. It is also involved in the survival and differentiation of cells, metastasis and in ECM remodeling (13,14). Periostin-deficient animal models demonstrate delayed wound repair (15) and periostin has been described as a novel pro-angiogenic factor leading to significant enhancement of angiogenesis in human breast, gastric and ovarian cancer (16,17). The acquired expression of periostin promotes tumor angiogenesis through upregulation in the expression of VEGFR2 (18).

Based on the evidence previously mentioned, the present study hypothesized that periostin is important in angiogenesis in keloid and, therefore, examined the expression of periostin in keloids and in normal skin and its association with blood vessel density. Subsequently, the present study investigated whether the periostin that is secreted by keloid fibroblasts (KFs) affects endothelial cell migration and angiogenesis and aimed to elucuidate the underlying mechanism *in vitro*. Furthermore, the association between periostin and other known angiogenic factors, including VEGF and angiopoietin-1 (Ang-1) were examined.

The article "Upregulated periostin promotes angiogenesis in keloids through activation of the ERK 1/2 and focal adhesion kinase pathways, as well as the upregulated expression of VEGF and angiopoietin-1" was published in 2014. Journal: Mol Med Rep.

## Materials and methods

The present study was performed in compliance with the regulations of the Medical Ethics Committee of Peking University Third Hospital, Beijing, China.

### Skin specimens and immunochemistry

Specimens of keloid tissue (n=15) and normal skin (n=11) were obtained from the discarded tissues of patients receiving plastic surgery to remove the keloid, following the provision of written informed consent. None of the patients (9–84 years old) had received treatment for the keloids prior to surgical excision.

The tissues were fixed in 4% paraformaldehyde, embedded in paraffin and mounted on glass slides. These were deparaffinized and immersed in 0.01 M citrate buffer (pH 6.0; Zhongshan Golden Bridge Biotechnology Co., Ltd., Beijing, China), heated in a microwave oven (Midea, Fushan, China), cooled for 30 min to room temperature and then washed in water. Endogenous peroxidase was inhibited using 3% H_2_O_2_. The slides were then incubated at 4°C overnight with a rabbit antibody against human periostin (1:100; ab14041; Abcam, Cambridge, MA, USA) or mouse antibody against human CD31 (1:80; ZM-0044) or CD105 (1:50; ZM-0297) from Zhongshan Golden Bridge Biotechnology Co., Ltd. Phosphate-buffered saline (PBS; Zhongshan Golden Bridge Biotechnology Co., Ltd.) was used as a negative control. The antibodies were diluted in 1% bovine serum albumin (BSA; Sigma, St. Louis, MO, USA)/Tris-buffered saline (Zhongshan Golden Bridge Biotechnology Co., Ltd.). Following washing, the slides were incubated with biotinylated anti-rabbit or anti-mouse immunoglobulin (Ig)G (Zhongshan Golden Bridge Biotechnology Co., Ltd.) secondary antibody (60 min at 37°C). Following washing with PBS, the slides were stained using a diaminobenzidine kit (Zhongshan Golden Bridge Biotechnology Co., Ltd.). Image-Pro Plus 6.0 (Media Cybernetics, Inc., Bethesda, MD, USA) was used for quantified analysis to calculate the integrated optical density of each antigen density.

### Primary cell culture and treatment

The KFs were isolated from the discarded keloid tissues obtained from the patients during surgery (n=6). All keloid tissues were obtained from untreated, primary lesions. The KFs were maintained in Dulbecco’s modified Eagle’s medium (DMEM; Gibco, Grand Island, NY, USA) supplemented with 10% fetal bovine serum (FBS; HyClone, Logan, UT, USA) containing 100 U/ml penicillin and 100 U/ml streptomycin (Invitrogen Life Technologies, Carlsbad, CA, USA). The KFs between passages 4 and 8 were used in the subsequent experiments. Primary human umbilical vein endothelial cells (HUVECs) were isolated from segments of the human umbilical cord vein by collagenase digestion and cultured in medium 199 (M199) supplemented with 10% FBS, as described previously (19). The subsequent experiments were conducted using cells at passages between 2 and 6.

The article "Upregulated periostin promotes angiogenesis in keloids through activation of the ERK 1/2 and focal adhesion kinase pathways, as well as the upregulated expression of VEGF and angiopoietin-1" was published in 2014. Journal: Mol Med Rep.

Recombinant human periostin protein (rhPN; BioVendor, Brno, Czech Republic) was treated with different concentrations (10, 50 and 100 ng/ml). For inhibitory studies, the cells were pretreated with 10 μM U1206 [extracellular signal-regulated kinase 1/2 (ERK1/2) inhibitor; Cell Signaling Technology, Beverly, MA, USA)] or 10 μM focal adhesion kinase (FAK) inhibitor 14 (Santa Cruz Biotechnology, Inc., Santa Cruz, CA, USA) for 1 h at 37°C. For knock down of periostin, the KFs were transfected with short hairpin RNA (shRNA; Genechem, Shanghai, China) against periostin, as previously described (20).

### Western blot analysis

The KFs were washed twice with ice-cold PBS and then harvested with lysis buffer (Beyotime, Shanghai, China) containing phosphatase and protease inhibitors. The protein concentration was quantified using a Bicinchoninic acid Protein Assay kit (CoWin Biotech, Beijing, China). The proteins in the lysates were separated using sodium dodecyl sulfate-polyacrylamide gel electrophoresis (SDS-PAGE; Beyotime) and were then transferred onto a nitrocellulose membrane (Applygen Technologies, Inc., Beijing, China), which was inhibited with 5% BSA at room temperature for 1 h. This was then incubated at 4°C overnight with the primary antibodies, anti-protein kinase B (Akt) (ab32038, rabbit monoclonal to Akt, 1:1,000) or anti-phospho-Akt [ab81283, rabbit monoclonal to Akt (S473), 1:1,000) (both purchased from Abcam, Cambridge, UK), anti-ERK1/2 (ab17942, rabbit polyclonal to ERK1 + ERK2, 1:1,000) or anti-phospho-ERK1/2 [ab76165, rabbit polyclonal to Erk1 (pT202/pY204) + Erk2 (pT185/pY187), 1:1,000] (both purchased from Epitomics, Cambridge, UK), anti-FAK (ab40794, rabbit monoclonal to FAK, 1:500) or anti-phospho-FAK [ab4803, rabbit polyclonal to FAK (phospho Y397), 1:500] (both purchased from Abcam), or anti-β-actin (TA-09, mouse monoclonal to β-actin; Zhongshan Golden Bridge Biotechnology, Inc.). This was followed with the corresponding IgG secondary antibody (1:10,000; LI-COR Biosciences, Lincoln, NE, USA) for 1 h away from light. All antibodies were anti-human. The membranes were then scanned using the Odyssey Infrared Imaging system (LI-COR Biosciences) to detect the expression quantity of each protein.

### Enzyme-linked immunosorbent assay (ELISA)

The secreted VEGF and Ang-1 were quantified using ELISA kits (Neobioscience Technology Co., Ltd., Beijing, China and Abcam, respectively). Briefly, the 96-well microplates were coated overnight with 100 μl capture antibody in a sealed bag at room temperature, washed three times with wash buffer, then inhibited with reagent diluent for 1 h. A 100 μl quantity of all standards and cell medium samples were added to the 96-well plate for incubation for 2 h. Following 2 h incubation with the detection antibody, 20 min incubation with a working dilution of horseradish peroxidase-conjugated streptavidin and 20 min incubation with the substrate solution in a light-resistant container, stop solution was added to each well. The absorbance was calculated at 450 nm, correcting for plate artifacts at 570 nm and a log-transformed standard curve.

The article "Upregulated periostin promotes angiogenesis in keloids through activation of the ERK 1/2 and focal adhesion kinase pathways, as well as the upregulated expression of VEGF and angiopoietin-1" was published in 2014. Journal: Mol Med Rep.

### Fibroblast-conditioned medium preparation

Cell-conditioned medium was harvested from the KFs or normal fibroblasts (NFs) 3 days following plating. These were centrifuged at 2×10^4^ rpm for 5 min to remove cellular debris and were stored at −20°C prior to the tube formation assay. Prior to performing the assays, the conditioned medium and M199 at 10% were mixed at a 1:1 ratio.

### Cell migration assay

The KFs that were incubated with DMEM with 0.1% FBS were seeded at 5×104/ml onto Transwell inserts (Millipore, Billerica, MA, USA) with an 8 μm pore-size membrane above 24-well plates and 600 μl DMEM with 10% FBS was added to each well. Following incubation for 24 h, the inserts were fixed with methanol for 15 min and washed with PBS prior to staining with 0.5% crystal violet solution (Sigma) for 30 min. The number of migrated cells was counted using phase-contrast microscopy (magnification, ×200). Six randomly selected fields were counted per insert.

### Tube formation assay

The 96-well plates were coated with 100 μl growth-factor-reduced Matrigel™ (BD Biosciences, San Jose, CA, USA), which was allowed to polymerize for 1 h at 37°C. The HUVECs (2×10^4^ cells/well), which were treated with different conditioned medium were seeded onto the Matrigel™. Tube formation and were assessed following 24 h incubation under an inverted phase contrast microscope (Olympus, Tokyo, Japan). The mean total length of the tube formed was determined using Image-Pro Plus software (Media Cybernetics LP, Silver Spring, MD, USA) in 6 randomly selected fields/well.

### Statistical analysis

Statistical analysis involved use of SPSS 12.0 (SPSS Inc., Chicago, IL, USA). Quantitative data are expressed as the mean ± standard deviation (SD) from at least three independent experiments. Pearson’s correlation test was used for correlative analysis. One-way ANOVA followed by Scheffe’s post-hoc test were used to compare multiple groups. P<0.05 indicated a statistically significant difference.

The article "Upregulated periostin promotes angiogenesis in keloids through activation of the ERK 1/2 and focal adhesion kinase pathways, as well as the upregulated expression of VEGF and angiopoietin-1" was published in 2014. Journal: Mol Med Rep.

## Results

### Periostin level is increased and correlated with blood vessel density in human keloid tissue

The expression of periostin and the vascular endothelial-cell markers CD31 and CD105 were examined using immunohistochemistry to examine whether the expression of periostin and the density of blood vessels differed between the keloid and the normal skin tissue. Periostin was expressed in the epidermis and dermis of the two tissues (Fig. 1A). The protein level of periostin was 2.3-fold higher in the keloid tissue compared with the normal skin (Fig. 1B). Blood vessel density, which was assessed by CD31 and CD105 staining, was 1.6- and 3.6-fold higher in the keloidtissue compared to the normal tissue, respectively (Fig. 1B). A marked positive correlation was observed between the level of periostin protein and the blood vessel density in the CD31 staining (r=0.711, P<0.01) and a weak correlation was observed following CD105 staining (r=0.251, P<0.01) in keloid tissue (Fig. 1C and D).

### Upregulated periostin in conditioned medium from KFs increases HUVEC migration and tube formation

To determine whether the periostin secreted by fibroblasts affected angiogenesis, the present study examined the migration and tube formation of HUVECs using conditioned medium from the KFs and NFs. Firstly, the KFs were transfected with either shRNA against periostin or control shRNA. Fluorescence microscopy and reverse transcription quantitative polymerase chain reaction (RT-qPCR) analyses were performed to ensure the efficiency of transfection prior to each experiment (Fig. 2). Use of the KF-conditioned medium significantly increased the number of migrating cells compared with the NF-conditioned medium (Fig. 3A). In addition, KF-conditioned medium promoted tube formation when compared with the NF-conditioned medium (Fig. 3B). Notably, the conditioned medium from the KFs with shRNA knock down of periostin significantly inhibited migration and tube formation compared with the controls. To exclude the effect of other factors in the conditioned medium, the effect of rhPN treatment at different concentrations on HUVEC migration and tube formation was examined. Contrary to the effects of conditioned medium from the KFs with shRNA periostin-knockdown, treatment with rhPN dose-dependently promoted migration (Fig. 4A) and tube formation (Fig. 4B).

### Periostin promotes HUVEC migration and tube formation by activating the ERK1/2 and FAK pathways

To clarify the mechanism of periostin-promoted angiogenesis, the present study examined the involvement of several intracellular signaling molecules, including FAK, Akt and ERK in the HUVECs following incubation with rhPN. Incubation with rhPN increased the phosphorylation of FAK and ERK (Fig. 5A). To demonstrate the involvement of FAK and ERK in periostin-promoted angiogenesis, capillary tube formation was examined following treatment with either FAK inhibitor 14 or ERK inhibitor (U0126) together with rhPN. Treatment with FAK inhibitor 14 or U0126 suppressed FAK and ERK activity, respectively. FAK inhibitor 14 and U0126 inhibited the periostin-promoted migration (Fig. 5B) and tube formation (Fig. 5C) of the HUVECs, which suggested that periostin-induced angiogenesis is mediated by ERK1/2 and FAK activity.

The article "Upregulated periostin promotes angiogenesis in keloids through activation of the ERK 1/2 and focal adhesion kinase pathways, as well as the upregulated expression of VEGF and angiopoietin-1" was published in 2014. Journal: Mol Med Rep.

### Periostin affects VEGF and Ang-1 secretion in KFs

To investigate whether periostin affected the expression of other pro-angiogenic factors, the present study examined the expression of two angiogenic factors, VEGF and Ang-1, in the KFs following treatment with rhPN. Treatment with rhPN dose-dependently promoted the secretion of VEGF in the KFs (Fig. 6A). The expression of Ang-1 was increased following treatment with 50 or 100 ng/ml rhPN, however no difference was observed with 10 ng/ml rhPN (Fig. 6B).

## Discussion

The presents study demonstrated that the level of periostin and blood vessel density were higher in human keloid tissue compared with normal tissue and a positive correlation was observed between periostin level and blood vessel density. In addition, the increased periostin level in the KFs promoted angiogenesis by increasing the migration and tube formation of HUVECs via the ERK1/2 and FAK signal pathways. Periostin also affected the expression of VEGF and Ang-1 in the KFs and periostin may be a promising therapeutic target for treatment of keloids and other angioproliferative diseases.

Although keloids are defined as a dermal benign disorder, their behavior resembles that of tumor cells, with keloids exhibiting biological characteristics of tumor cells, including bioenergetics, hyperproliferation and invasion (21,22). The induction of angiogenesis is considered important in the cascade of tumor invasion (23). To maintain the invasive characteristics and ability to recur, tumor-like keloids require the generation of numerous new blood vessels to maintain a steady supply of oxygen and nutrients. The histological characteristics of keloids also demonstrate tumor properties. In general, keloids can be divided into three areas, which exhibit distinct histological features: a central stable portion, an erythematous border and a normal skin periphery (1,22). The central stable portion features a local state of hypoxia due to the overproliferation of endothelial cells and the deposition of abundant collagen leading to capillary occlusion. The border contains proliferative fibroblasts and an increased density of blood vessels, which invade the peripheral normal skin. In the present study, blood vessel density, examined by staining with CD31 and CD105, was greater in the keloid tissues compared with the normal tissues, consistent with previous studies by Amadeu *et al* (24) and Appleton *et al* (25). CD31 and CD105 are endothelial antigens, which have been used as direct markers of the degree of neoangiogenesis. In the present study, the increased periostin level in keloids was correlated with the expression of CD31 and CD105, which suggested that periostin may promote angiogenesis in keloids.

The article "Upregulated periostin promotes angiogenesis in keloids through activation of the ERK 1/2 and focal adhesion kinase pathways, as well as the upregulated expression of VEGF and angiopoietin-1" was published in 2014. Journal: Mol Med Rep.

Fibroblasts are responsible for the construction and remodeling of extracellular components and angiogenesis is an essential process in the progression of keloids (19,25). Previous studies have demonstrated that several growth factors and cytokines are regulated in KFs and certain types, including VEGF and TGF-β, promote angiogenesis in keloids (5). The present study revealed that the synthesis and secretion of periostin was greater in the KFs compared with the NFs. Conditioned medium from KFs promoted the migration and tube formation of HUVECs and rhPN promoted angiogenesis in a dose-dependent manner. Notably, knock down of periostin decreased the HUVEC migration and angiogenesis stimulated by the conditioned medium. Periostin promotes the survival of endothelial cells and angiogenesis in certain types of cancer and angiogenesis and lymphangiogenesis have been observed to correlate with periostin in non-small cell lung cancer (26). Additionally, acquired periostin in breast cancer promotes tumor angiogenesis by upregulating the expression of endothelial growth factor receptor 2 (18) and use of a periostin antibody significantly inhibits tumor growth and angiogenesis *in vivo* (27). Therefore, periostin promotes angiogenesis to directly affect the development of keloids and is, therefore, a novel pro-angiogenic factor involved in angiogenesis in keloids.

The present study examined the possible mechanism underlying the action of periostin in endothelial cells. Previous studies revealed that growth factors stimulate angiogenesis via activating kinase signaling pathways, including PI3K/AKT, ERK1/2, FAK and p38/MAPK, to regulate endothelial cell migration, survival and vascular permeability (28,29). In the present study, periostin promoted HUVEC migration and tube formation by activating the ERK1/2 and FAK pathways. The ERK pathway is activated by various stimuli, including mitogen kinases and cell survival factors and also regulates the cell cycle of endothelial cells. FAK is a cytoplasmic tyrosine kinase, which is important in integrin-mediated signal transduction. Upregulation in its expression has been observed in several cancer cells and it is important in tumor angiogenic activity and progression (30). The interaction between periostin and integrin triggers intracellular signaling, which promotes the tube formation and migration of lymphatic endothelial cells during lymphangiogenesis (26). The results of the present study demonstrated that treatment with either ERK1/2 or FAK inhibitors reduced the migration and tube formation of HUVECs, which suggested that the periostin-activated ERK1/2 and FAK pathways are involved in angiogenesis.

The article "Upregulated periostin promotes angiogenesis in keloids through activation of the ERK 1/2 and focal adhesion kinase pathways, as well as the upregulated expression of VEGF and angiopoietin-1" was published in 2014. Journal: Mol Med Rep.

Regulation of angiogenesis in keloids is complex and is controlled by a variety of pro-angiogenic factors. VEGF is the most potent angiogenic factor due to its high specificity to endothelial cells (31). It is closely associated with keloid pathogenesis. Previous studies have demonstrated that VEGF production is abundant in the underlying dermis of keloids and that the expression of VEGF is higher in keloid-derived fibroblasts compared with normal skin fibroblasts *in vitro* (5). In the present study, periostin promoted the secretion of VEGF in the KFs, which was similar to its expression in periodontal ligament cells and lymphatic endothelial cells. Ang-1, a main ligand for Tie2, is an angiogenic growth factor that specifically functions to induce endothelial migration, tube formation and survival (32). In addition, Ang-1 acts to cooperatively stimulate VEGF, which accelerates the closure of endothelial cell scratch-wounds. The present study also found that periostin increased the expression of Ang-1 in the KFs and periostin may indirectly promote angiogenesis by increasing the expression of VEGF and Ang-1.

Appropriate regulation of periostin is required throughout the repair process as dysregulation of periostin leads to excess proliferation, including the formation of hypertrophic scars and keloids or even tumors. Our previous study found that periostin was highly expressed in keloids and gradually increased between normal skin and hypertrophic scars to keloids (11). Accumulating evidence indicates that the expression of periostin is positively correlated with tumor grade and stage in several types of tumor, including hepatocellular carcinoma, colorectal cancer and prostate cancer (33,34). The results of the present study demonstrated that periostin-induced angiogenesis underlies the pathology of keloids and the level of periostin may affect the process of hyperplasia and regression.

In conclusion, the present study revealed that the expression of periostin was increased in human keloid tissue and correlated with blood vessel density. The upregulated level of periostin promoted angiogenesis by activating the ERK1/2 and FAK signaling pathways and increasing the secretion of VEGF and Ang-1. Therefore, periostin may promote angiogenesis in keloids and be a key factor in their development. These findings may contribute to an improved understanding of keloid pathogenesis and may provide a novel therapeutic target in the treatment of keloids and other angioproliferative diseases.

The article "Upregulated periostin promotes angiogenesis in keloids through activation of the ERK 1/2 and focal adhesion kinase pathways, as well as the upregulated expression of VEGF and angiopoietin-1" was published in 2014. Journal: Mol Med Rep.

## Figures and Tables

**Figure 1:** Periostin and blood vessel density are higher in keloid tissue compared with normal skin tissue. (A) Immunohistochemical staining of periostin, CD105 and CD31 in keloid and normal tissues. (A and B) Level of periostin in normal skin and (C and D) keloid tissue. (E and D) Level of CD31 in normal skin and (G and H) keloid tissue. (I and J) CD105 in normal skin and (K and L) keloid tissue (arrows indicate blood vessels). (B) Changes in integrated optical density in the expression of periostin, CD105 and CD31 for all groups. (C and D) Spearman correlation analysis was performed to analyze correlations between the expression of periostin and the expression of (C) CD31 or (D) CD105 in the keloid tissues. ^*^P<0.05 and ^**^P<0.01, compared with the controls.

**Figure 2:** Lentiviral-mediated stable genetic knockdown in KFs. KFs were transfected with lentivirus harboring shRNA periostin or non-silencing shRNA. (A) Fluorescence microscopy of sh-pn under (a) microscopy and (b) fluorescence microscopy; non-silencing group under (c) microscopy and (d) fluorescence microscopy. (B) mRNA analyses were performed to ensure the efficiency of transfection prior to each experiment (n=6). ^*^P<0.05, compared with the controls. n.s,, not significant; KF, keloid fibroblasts; shRNA, short hairpin RNA; sh-pm, shRNA-periostin; NC, non-silencing.

**Figure 3:** Upregulated periostin in CM from KFs increases HUVEC (arrow) migration and tube formation compared with the NFs. (A) Migration and (B) tube formation of HUVECs in (a) NF-CM, (b) KF-CM, (c) sh-nc KF-CM and (d) sh-pn KF-CM. (n=6). n.s., not significant; CM, conditioned medium; KF, keloid fibroblasts; HUVEC, human umbilical vein endothelial cell; NF, normal fibroblasts; sh-nc KF, KFs with non-silencing short hairpin RNA; sh-pn KF, KFs with short hairpin RNA against periostin.

**Figure 4:** rhPN promotes HUVEC migration and tube formation. (A) Migration and (B) tube formation of HUVECs following treatment with rhPN: (b) 10 ng/ml, (c) 50 ng/ml, (d) 100 ng/ml and (a) a negative control of albumin without rhPN. ^*^P<0.05 and ^**^P<0.01. (n=6). rhPN, recombinant human periostin protein; HUVEC, human umbilical vein endothelial cell.

The article "Upregulated periostin promotes angiogenesis in keloids through activation of the ERK 1/2 and focal adhesion kinase pathways, as well as the upregulated expression of VEGF and angiopoietin-1" was published in 2014. Journal: Mol Med Rep.

**Figure 5:** Periostin promotes HUVEC migration and tube formation by activating the ERK1/2 and FAK pathways. (A) Western blot analysis of the phosphorylation of Akt, ERK1/2 and FAK in HUVECs treated with 50 ng/ml rhPN for the indicated time periods. (B) Migration and (C) tube formation of HUVECs (arrow) treated (a) without rhPN as a control and with (b) 50 ng/ml rhPN, (c) rhPN and ERK1/2 inhibitor U1206 or FAK inhibitor for 14 days. ^**^P<0.01. (n=6). HUVEC, human umbilical vein endothelial cell; p-, phosphorylated; ERK1/2, extracellular signal-regulated kinase 1/2; FAK, focal adhesion kinase; Akt; protein kinase B; rhPN, recombinant human periostin protein.

**Figure 6:** Periostin promotes VEGF and Ang-1 secretion in KFs. KFs were treated with or without rhPN at different concentrations (0, 10, 50 and 100 ng/ml). (A) Enzyme-linked immunosorbent assay of the expression of VEGF and (B) Ang-1 in the KF supernatant. Data are presented as the mean ± standard deviation from at least three independent experiments. ^*^P<0.05 and ^**^P<0.01.(n=6). n.s., not significant; VEGF, vascular endothelial growth factor; Ang-1, angiopoietin-1; KF, keloid fibroblasts; rhPN, recombinant human periostin protein.
